# Study on the Mechanism of miR-146a in Gingival Mesenchymal Stem Cells

**DOI:** 10.1155/2022/1630260

**Published:** 2022-11-15

**Authors:** Fang Wang, Zheng Jing, Ting Wei, Hui Jiang, Xiaojun Li

**Affiliations:** ^1^Stomatology Hospital, School of Stomatology, Zhejiang University School of Medicine, Zhejiang Provincial Clinical Research Center for Oral Diseases, Key Laboratory of Oral Biomedical Research of Zhejiang Province, Cancer Center of Zhejiang University, Hangzhou 310006, China; ^2^Department of Periodontology, the Affiliated Stomatology Hospital, Zhejiang University School of Medicine, Hangzhou 310006, China; ^3^Central Hospital of Haining, Jiaxing 314408, China

## Abstract

This study aimed to investigate the molecular mechanisms of microRNA-146a (miR-146a) on gingival mesenchymal stem cells (MSCs). Gingival MSCs were isolated from the gingiva tissues of patients with periodontal disease to reveal the function of miR-146a in regulating osteoblast differentiation. miR-146a inhibits osteoblast differentiation by inhibiting phosphorylated cyclic-AMP response binding (CREB) protein translocation into the nucleus and ultimately attenuating runt-related transcription factor 2 (Runx2) expression. Furthermore, silencing miR-146a promotes the proliferation of gingival MSCs. Of note, targeted inhibition of miR-146a also inhibited LPS-induced inflammatory response and promoted the proliferation of gingival MSCs via CREB/Runx2 axis. MiR-146a is a key negative regulator of gingival MSCs proliferation and osteogenic differentiation, and targeting to reduce the miR-146a expression is essential for bone formation signaling. Therefore, we propose that miR-146a is a useful therapeutic target for the development of bone anabolic strategies.

## 1. Introduction

Periodontal disease is the most common oral disease, including categories of gum disease and periodontitis with deep periodontal tissue lesions, considered to be the main cause of tooth loss in adults, as well as the most significant oral disease that endangers human dental and even systemic health [1]. Periodontitis is mainly a chronic inflammatory disease of periodontal supporting tissues caused by bacteria and is highly prevalent worldwide [2, 3]. Currently, the promotion of dental bone and alveolar bone regeneration is considered to be the most promising treatment strategy for periodontitis [4, 5]. Remodeling periodontal connective tissue and promoting bone and alveolar bone regeneration have been considered the most promising treatment strategy for periodontitis. Unfortunately, due to the complexity and specificity of the pathogenesis of periodontitis and the periodontal microenvironment, conventional treatments are unable to completely repair the periodontal tissue damage caused by periodontitis [6]. Notably, with the maturation of stem cell and biological tissue engineering technologies (e.g., guided tissue regeneration, GTR), stem cells, especially periodontal stem cells, were considered to be the most reliable method to promote dental bone regeneration for the treatment of periodontitis and an important link to identify ideal seed cells [7].

As a primitive cell population with self-renewal and multidirectional differentiation potential, MSCs, the cells of origin for the formation of various tissues and organs, have emerged as effective alternative cell sources for tissue engineering. Stem cells from the bone marrow and dental marrow have been shown to have a role in promoting periodontal osteogenesis [8, 9]. Dental-derived MSCs were extracted from the dentition and its accessory tissues. However, these MSCs are usually limited in their general application by the small number of dental-derived MSCs, the invasive process of obtaining them, and the difficulty of their proliferation and differentiation *in vitro*. Therefore, gingiva MSCs, which have properties easily obtained *via* minimally invasive cell isolation techniques, phenotypic stability, and multidirectional differentiation potential, have attracted wide attention in the application of periodontal disease prevention and treatment. Numerous studies have shown that gingiva MSCs are crucial for tissue regeneration and immunomodulation, and their ability to promote periodontal bone regeneration has been demonstrated in animal models [10, 11].

MicroRNA (miRNA), a class of small noncoding RNA sequences consisting of approximately 22 nucleotides, can regulate eukaryotic gene expression and influence the synthesis of proteins encoded by target genes, thus participating in almost all cellular life activities, including cell proliferation, differentiation, metabolism, immune regulation, inflammatory response, and cell death. Numerous studies implied that miRNAs have played key roles in various aspects of periodontal tissue injury and repair, inflammatory response, and homeostasis of the periodontal microenvironment, including promoting periodontal stem cell differentiation and regulating osteoblast and osteoclast functions [12, 13].

Previously, miR-146a, miR-143-3p, and miR-1226 have been reported to be positively associated with the progression of chronic periodontitis as well as other periodontal diseases [14, 15]. Previous studies showed that miR-146a could promote angiogenesis in human umbilical vein endothelial cells (PMID: 28337286), regulate the function of Th17 cell differentiation to modulate cervical cancer cell growth and apoptosis (PMID: 30864722) and mitochondrial function, and cardiomyocyte apoptosis (PMID: 33717647). In addition, miR-146a negatively regulates osteogenesis and bone regeneration in adipose-derived mesenchymal stem cells (PMID: 28205638). Of particular note, miR-146a has been shown to be a potential therapeutic target for chronic periodontitis by inhibiting the chronic inflammatory response and immunomodulatory effects of periodontal tissues [17]. However, the role and molecular basis of miR-146a-regulated osteogenic differentiation of gingiva MSCs remain unclear, which greatly limits its clinical application and transformation as a therapeutic target. Here, we mechanically evaluated the effects of miR-146a on cell proliferation and osteogenesis of gingiva MSCs. Our findings suggest that miR-146a plays a pivotal role in gingival mesenchymal stem cell proliferation and osteogenic differentiation. Thus, targeting to reduce the miR-146a expression is essential for bone formation signaling, which may be a new early warning and therapeutic target for chronic periodontitis.

## 2. Materials and Methods

### 2.1. Reagents

Minimum Essential Medium *α* (*α*-MEM) and fetal bovine serum (FBS) were bought from HyClone (Logan, Utah, USA). Cell Counting Kit-8 (CCK-8) kit was obtained from Dojindo Laboratories (Kumamoto, Japan). Cell Cycle and Apoptosis Analysis Kit were obtained from Beyotime Biotechnology (Shanghai, China). The Oil Red O staining Kit was obtained from Solarbio Science and Technology Co., Ltd. (Beijing, China). MiR-146a inhibitor and miR-146a mimics were obtained from Shanghai GenePharma Co., Ltd. All other chemicals were of analytical grade.

### 2.2. Gingiva MSCs Isolation and Culture

The gingiva was obtained from patients with periodontal diseases. The volunteers were admitted to the periodontal department of the Zijingang branch of the affiliated stomatology hospital, Zhejiang University School of Medicine. All procedures are approved by the clinical research ethics committee of Zhejiang University School of medicine and informed consent was provided 2021-88 (R). The gingiva MSCs were isolated and cultured as previously described [18]. Gingiva MSCs were cultured in *α*-MEM with 15% fetal bovine serum (FBS) supplemented with 1% (v/v) penicillin and streptomycin in a constant environment of 37°C/5% CO_2_. All cells were harvested after specific treatments for further investigation.

### 2.3. Flow Cytometric Analysis

We sorted MSCs by flow cytometry based on their expressed surface markers of CD29, CD90, and CD105, not CD34. Gingiva MSCs were stained with specific phycoerythrin (PE) conjugated anti-human CD29 and CD105 (BioLegend), CD34 (eBioscience, Thermo Fisher Scientific), CD90 (R&D Systems) antibodies. Flow cytometry data were analyzed using CellQuest analysis software (BD Biosciences). Cell cycle and apoptosis assays were also completed by flow cytometry.

### 2.4. Adipogenic Differentiation

Gingiva MSCs were planted on 6-well plates with the *α*-MEM growth medium and allowed to adhere overnight. Then, the medium was changed to DMEM medium containing 10% FCS, 1 *μ*M dexamethasone (Sigma), 200 *μ*M indomethacin (Sigma), 10 *μ*M insulin (Sigma), 0.5 mM isobutyl-methylxanthine (IBMX, Sigma) and 1% antibiotic/antimycotic. After 2 weeks, the formation of oil globules was determined through Oil Red O staining.

### 2.5. Infection of miR-146a Overexpression

We insert miR-146a and sponge sequence into a pLVX-H1-GFP-puro cloning vector (GenePharma) to generate lentivirus. The PCR primers are provided in Supplementary Table 2. Transfection of gingiva MSCs with the plasmid of miR-146a overexpression and sponge to receive lentivirus for the subsequent experiment [19]. The transfection effect was observed using fluorescence microscopy [20].

### 2.6. Gingiva MSCs Viability Test

Gingiva MSCs were seeded in 96-well plates with 4 × 10^3^ cells/well. Gingiva MSCs were transfected with miR-146a overexpressing lentivirus and cultured continuously for 7 days, and cells transfected with an overexpressing empty plasmid were used as control. The proliferation activity of gingiva MSCs was detected daily using a flat plate clone formation test and CCK-8 assay according to the vendor's instructions.

### 2.7. Osteoblast and Osteoclast Differentiation

Gingiva MSCs plated in 6-well plates were maintained in an *α*-MEM medium containing 10% FBS, 10 mM dexamethasone (Sigma), and 10 mM *β*-glycerophosphate (Alfa Aesar), 50 *μ*M Vitamin C (Sigma) and 1% antibiotic/antimycotic. Gingiva MSCs were continuously cultured for 4 weeks before applying von Kossa staining to detect mineralized nodules. Medium changes are done every 4 days during the culture. Meanwhile, gingiva MSCs were cultured in *α*-MEM containing 10% FBS and 50 ng/ml RANKL (R&D), and 25 ng/ml M-CSF (Peprotech) to assay the osteoclastogenesis. After 10 days of culture, the gingiva MSCs were subjected to PBS wash and then fixed in 4% paraformaldehyde solution for 10 minutes before TRAP (anti-tartrate acid phosphatase) staining, and finally observed under an inverted microscope. Osteoblasts and osteoclast were cocultured with the miR-146a overexpression plasmid in 6-well plates for 7 days, respectively. Subsequently, the expression levels of relevant genes and proteins in osteoblasts and osteoclasts were measured.

### 2.8. Quantitative Real-Time PCR

To further verify the results, real-time PCR was employed to quantify relative mRNA expression levels. First, the mRNA was extracted from cells by Trizol (TAKATA, Osaka, Japan) and reverse-transcriptional reactions were performed using a TAKATA Reverse Transcriptase kit (TAKATA, Osaka, Japan). Removal of DNase and cDNA reverse synthesis and real-time PCR were then performed as protocol. The qPCR reaction mixture was prepared using SYBR Green Master Mix (Tiangen, Beijing, China) and then run on a CFX ConnectTM Real-Time PCR System (Bio-Rad, California, USA) as previously described. U6 snRNA was used as an internal reference for miR-146a. GAPDH was used as an internal control for other gene assays in this study. The qPCR primers are provided in Supplementary Table 2.

### 2.9. Western Blot

Western blot was commonly used to detect the protein expression level of cells. In short, proteins to be tested were extracted from cells and were separated within SDS- polyacrylamide gel electrophoresis (SDS-PAGE), then transferred into the polyvinylidene fluoride (PVDF) membranes. After blocking and incubation of corresponding antibodies (Supplementary Table 1) for 12 h, specific binding with second antibodies was performed, and the immunoblotting of target protein bands were observed using a ECL chemiluminescence and gel documentation system (G: BOX F3, Gene).

### 2.10. Statistical Analysis

All data were expressed as the Mean ± S.D. Statistical analysis was performed using GraphPad Prism 8.0 Software (San Diego, CA, USA). Comparisons between two groups and among three or more groups were achieved using the two-tailed unpaired *t*-test or analysis of variance (ANOVA), respectively. *P* < 0.05 was considered statistically significant.

## 3. Results

### 3.1. Characterization of Gingiva MSCs from Gingiva with Periodontitis

Macroscopically, gingiva MSCs from gingiva with periodontitis appeared with a spindle fibroblast-like morphology under light microscopy, similar to other types of MSCs (Figure 1(a)). Subsequently, the abundance of surface markers in gingiva MSCs was determined by flow cytometry and immunofluorescence. As shown in Figure 1(b), CD29, CD105, and CD90 showed a positive expression and CD34 showed negative expression in gingiva MSCs. Meanwhile, we used Oil Red O staining to test the differentiation potential of gingiva MSCs. Moreover, lipid accumulation was observed in the cytoplasm of those differentiated gingiva MSCs after 2 weeks of culture in a lipogenic differentiation medium, indicating existed differentiated gingiva MSCs (Figure 1(c)). In contrast, no positive signals were observed in the cells cultured with the standard medium. These results confirm that cultured gingiva MSCs from gingiva with periodontitis possess stem cell properties.

### 3.2. miR-146a Affected the Proliferation of Gingiva MSCs

Gingiva MSCs were infected with lentiviruses carrying either a pLVX-H1-GFP-miR-146a or pLVX-H1-GFP-miR-146a-sponge plasmid. Stably transfected cells show bright green fluorescence (Figure 2(a)). Meanwhile, the miR-146a expression level was significantly elevated after pLVX-H1-GFP-miR-146a transfection, while pLVX-H1-GFP-miR-146a-sponge plasmid transfection was able to significantly attenuate the expression level of miR-146a in gingiva MSCs (Figure 2(b)). Cell proliferation viability assay by CCK-8 method showed that overexpressed miR-146a had a significant inhibitory effect on gingiva MSCs growth, in contrast, silencing miR-146a promotes gingiva MSCs proliferation (Figure 2(c)). The inhibition of miR-146a was found to significantly promote gingiva MSCs colony formation by clonogenic assay than normal and/or miR-146a overexpressed gingiva MSCs (Figure 2(d)). Notably, the results of cell cycle and apoptosis assays indicated that the overexpression of miR-146a profoundly reduced the proliferative viability of gingiva MSCs with concomitant effects on cell survival (Figures 2(e) and 2(f)), which suggested that miR-146a likely acted as a key factor affecting the proliferation of gingiva MSCs.

### 3.3. Silencing miR-146a Attenuates LPS-Mediated Inflammatory Response in Gingiva MSCs

Chronic inflammation of the periodontal tissue from the deep gingival layer to the periodontium and alveolar bone is a key factor in triggering periodontitis [21]. Inflammatory factors released by periodontal tissue cells, such as TNF-*α*, IL-6, and IL-1*β*, maintain the periodontal inflammatory environment for a long time and can lead to irreversible periodontal tissue damage [22]. Therefore, we further assessed the regulatory role of miR-146a on the inflammatory response of gingiva MSCs. First, we examined the content and expression levels of inflammatory factors in gingiva MSCs overexpressing miR-146a. The results show that elevated miR-146a significantly promotes the secretion of inflammatory factors (Figures 3(a)–3(c)), and also increases the mRNA levels of TNF-*α*, IL-6, and IL-1*β* in gingiva MSCs (Figure 3(d)). Studies reveal that local inflammatory responses can exacerbate periodontal tissue damage and accelerate the progression of periodontitis [21]. Notably, silencing miR-146a in the LPS-mediated inflammatory response model of gingiva MSCs significantly decreased the mRNA and protein abundance of inflammatory factors and reduced their release (Figures 3(e)–3(h)). These data suggest that miR-146a can drive the inflammatory response in gingiva MSCs.

### 3.4. Effects of miR-146a on the Osteogenic Differentiation of Gingiva MSCs

The promotion of osteogenic differentiation of MSCs is considered the most promising therapeutic strategy for chronic damaging diseases of bone tissue in clinical settings, such as osteoporosis and osteoarthritis. As shown in Figure 4(a), gingiva MSCs were cultured for 4 weeks, and mineralized nodules were visualized using von Kossa staining after transfection with a control plasmid, but not visualized with miR-146a overexpression plasmid. Cells were cultured in the medium for osteoclasts for 10 days and osteoclast was detected by TRAP staining. Similarly, TRAP-positive staining was observed in cells after transfected with a control plasmid but was almost not visualized with the miR-146a overexpression plasmid. Meanwhile, the result of coculture showed that miR-146a significantly decreased the expression of several core binding factors of osteogenic differentiation in hepatocytes, including bone morphogenetic protein 2 (BMP2), alkaline phosphatase (ALP), collagen type I collagen *α*1 (COL1*α*1), osteopontin (OPN), and osteocalcin (OCN) (Figure 4(b)). Consistently, miR-146a severely reduced the expression levels of the osteogenic key proteins (BMP2, COL1*α*1, OPN, and OCN) in gingiva MSCs. Briefly, these data indicated that miR-146a can inhibit osteogenic key enzyme expression to suppress osteogenesis in gingiva MSCs (Figures 4(c) and 4(d)).

### 3.5. miR-146a Regulates Osteogenesis in Gingiva MSCs *via* the CREB/Runx2 Axis

cAMP-response element-binding protein (CREB), an important transcriptional regulator, effectively promotes the osteogenic differentiation of MSCs [23]. Analyzing the interaction of miR-146a with target genes by target prediction database miRDB and miRcode, we found that CREB strongly interacts with miR-146a (Figure 5(a)). By overexpressing and/or silencing miR-146a, we confirmed that the expression of CREB is modified by miR-146a which in turn regulates osteogenesis in gingiva MSCs. Runt-related transcription factor 2 (Runx2) was a crucial regulator in promoting bone formation, which has important regulatory roles in osteoblast differentiation, chondrocyte maturation, and bone metabolism. First, we found that the overexpression of miR146 significantly attenuated CRBE/RUNX2-mediated osteogenic signaling in gingiva MSCs (Figures 5(b) and 5(c)). However, the overexpression of CREB was able to promote RUNX2 transcriptional regulation to restore miR-146a-mediated reduction in osteogenic key factor expression (Figures 5(d)–5(f)). These results reveal that miR-146a inhibits the osteogenic potential of gingiva MSCs *in vitro* by regulating the CREB/Runx2 axis.

## 4. Discussion

The osteogenic capacity of seed cells is an important indicator of periodontal tissue regeneration. Promoting the osteogenic potential of seed cells has been considered an important tool for periodontal osteogenesis and remodeling the physiological barrier of periodontal tissues [24]. With the advancement of tissue engineering technology, MSCs are widely used in clinical applications. Even though MSCs have multiple sources, gingiva MSCs have more distinct advantages due to their easy availability during routine dental procedures and the absence of significant differences in the characteristics of gingiva MSCs from healthy gingival tissues and those from hyperplastic or inflamed gingival tissues [25]. It has been shown that MSCs characteristics isolated from gingival tissues can exhibit a stable phenotype and have the potential for multidirectional differentiation during long-term culture [26]. Recent epidemiological surveys show that more than half of adults worldwide suffer from gingivitis and periodontitis, with a trend toward younger adults [27]. Clinically, the main goal of periodontitis treatment is to inhibit plaque and eliminate inflammation to prevent deterioration and recurrence of the disease [28]. Given the potential for directed differentiation of MSCs, using gingiva MSCs was expected to be an effective solution for the radical treatment of periodontitis [29]. Our previous study confirmed the osteogenic ability of gingiva MSCs, but the amount of new bone in rat bone defects was limited [26], so we tried to explore effective avenues to improve the osteogenic ability of gingiva MSCs and elucidate the molecular mechanism in this study.

MicroRNA, a noncoding single-stranded RNA regulated by posttranscriptional gene expression, plays an extremely important role in the inflammatory response, immune response, and almost all aspects of periodontal tissue, including periodontal stem cell differentiation, osteoblast function, and osteoclast function [30, 31]. miR-146a is one of the first miRNAs identified to be involved in the inflammatory response and is abnormally and significantly highly expressed in periodontal inflammatory tissues, promoting the development of periodontitis [31]. miR-146a has been reported to promote differentiation in periodontal ligament cells through the downregulation of NF-kappa B signaling (PMID: 20110513). In this study, we demonstrated that highly expressed miR-146a in periodontitis patient-derived gingiva MSCs can impair their osteogenic potential, block the cycle distribution of gingiva MSCs, and induce apoptosis. Similarly, the miR-146a overexpression drove inflammatory factor release in gingiva MSCs mediating the onset of inflammatory responses, and targeted inhibition of miR-146a significantly attenuated LPS-mediated inflammatory responses in gingiva MSCs. Interestingly, the targeted intervention of miR-146a activates Runx2 transcriptional regulation of the expression of key proteins (BMP2, OPN, OC, and BSP) of osteogenic signaling. Runx2 directly stimulates the transcription of osteocalcin, type I collagen, bone-bridging protein, and collagenase 3 genes to promote osteogenic differentiation during the differentiation of bone marrow mesenchymal cells to osteoblasts [32]. Bone morphogenetic protein (BMP), a target gene of Runx2 transcriptional regulation, is the most effective inducer of osteoblast differentiation and bone formation to regulate osteogenic differentiation [33]. BMP promotes osteogenic differentiation mainly by binding to heteromeric receptor complexes [34]. Evidence suggests that CREB is recruited to CRE in the Sma6 promoter and enhances the Smad6 expression and thus CREB regulates RUNX2 transcriptional activation was an important pathway to promote osteogenic differentiation [35]. As a “bridge” between the bone system and immune system, the CREB/Runx2 axis is a key factor to determine alveolar bone resorption or regeneration in the process of periodontitis development, and to a large extent affects the prognosis and outcome of periodontitis. To further elucidate the molecular mechanism of miR-146a regulation of Runx2, we predicted CREB as a potential target gene of miR-146a through the target gene database and performed validation. In this series of experiments, we demonstrated that miR-146a inhibits osteoblast differentiation by inhibiting phosphorylated CREB translocation into the nucleus and ultimately attenuating the Runx2 expression. These results suggest that targeted intervention of miR-146a to activate the CREB/Runx2 axis can promote osteogenesis and alleviate inflammation in gingiva MSCs.

Although this article also has some limitations. For example, CREB, as the predictive targeting gene, has not been validated by luciferase reporter assay. In addition, whether the same mechanism occurs in animal models of periodontitis or even in the periodontitis population remains to be answered. In follow-up studies, we will further verify the results of the study in vivo through animal model tests. Also, we know that most inflammatory mediators are produced by macrophages in the inflammatory environment. MSCs have been reported to skew LPS-stimulated macrophage polarization towards the M2-like phenotype and reduce inflammatory reactions by secreting TGF-*β* cytokines (PMID:31771622). However, whether the effect of miR-146a on inflammation is caused by macrophage polarization needs to be further investigated.

## 5. Conclusion

In summary, our findings suggest that miR-146a plays an important role in the osteogenic differentiation of gingiva MSCs through the CREB/Runx2 axis. miR-146a is a key negative regulator of gingival mesenchymal stem cell proliferation and osteogenic differentiation and targeting to reduce miR-146a expression is essential for bone formation signaling. Therefore, we propose that miR-146a holds promise as an attractive therapeutic target for periodontitis treatment.

## Figures and Tables

**Figure 1:** Characterization of gingiva MSCs from gingiva with periodontitis. (a). Gingiva MSCs morphology. (b). The abundance of surface markers in gingiva MSCs was determined by flow cytometry. (c). Oil Red O staining was used to test differentiated gingiva MSCs, the right panel were cells cultured with lipogenic differentiation medium, and the left panel with the standard medium.

**Figure 2:** miR-146a affected the proliferation of gingiva MSCs. (a) Detection of lentivirus carrying either a pLVX-H1-GFP-miR-146a or pLVX-H1-GFP-miR-146a-sponge plasmid infection, scar bar = 50 *μ*m. (b) Detection of the miR-146a expression level. (c) The effect of miR-146a on gingiva MSCs proliferation viability was tested by CCK-8. (d) The effect of miR-146a on Gingiva MSCs clonogenic viability was tested by colony formation assay. (e and f) Detection of cell survival by flow cytometry.

**Figure 3:** Silencing miR-146a attenuates the LPS-mediated inflammatory response in gingiva MSCs. (a–c) The content and expression levels of inflammatory factors in gingiva MSCs were tested. (d) The mRNA content of inflammatory factors in gingiva MSCs were tested. (c) The effect of miR-146a on Gingiva MSCs proliferation viability was tested by CCK-8. (e–h). silencing miR-146a in the LPS-mediated inflammatory response model of gingiva MSCs significantly decreased the mRNA and protein abundance of inflammatory factors and reduced their release.

**Figure 4:** Effects of miR-146a on the osteogenic differentiation of gingiva MSCs. (a) Mineralized nodules were visualized using von Cossa staining and osteoclast was detected by TRAP staining, the right panel is cells transfected with miR-146a overexpression plasmid, and the left panel with a control plasmid, scar bar = 50 *μ*m. (b) The mRNA content of BMP2, ALP, COL1*α*1, OPN, and OCN was tested. (c, d) BMP2, COL1*α*1,OPN, and OCN were tested by WB.

**Figure 5:** miR-146a regulates osteogenesis in gingiva MSCs via the CREB/Runx2 axis. (a) Analysis of the interaction of miR-146a with target genes by target prediction database. (b, c) CREB and Runx2 were tested by western blotting. (d–f) Osteogenic key factors expression was tested.

## Data Availability

The data and materials used to support the findings of this study are available from the corresponding author upon request.

## Supplementary Materials

Supplementary Materials Supplementary Table 1. List of the primary antibodies used for Western blotting (WB). Supplementary Table 2. Sequences of polymerase chain reaction (PCR) primer used in real-time PCR.
